# A Distinguishable Pseudo-Feature Synthesis Method for Generalized Zero-Shot Learning

**DOI:** 10.1155/2022/6220501

**Published:** 2022-11-29

**Authors:** Yunpeng Jia, Xiufen Ye, Yusong Liu, Huiming Xing, Shuxiang Guo

**Affiliations:** ^1^College of Intelligent Systems Science and Engineering, Harbin Engineering University, Harbin, Heilongjiang 150001, China; ^2^Faculty of Engineering, Kagawa University, Takamatsu, Kagawa 7608521, Japan

## Abstract

Generalized zero-shot learning (GZSL) aims to classify seen classes and unseen classes that are disjoint simultaneously. Hybrid approaches based on pseudo-feature synthesis are currently the most popular among GZSL methods. However, they suffer from problems of negative transfer and low-quality class discriminability, causing poor classification accuracy. To address them, we propose a novel GZSL method of distinguishable pseudo-feature synthesis (DPFS). The DPFS model can provide high-quality distinguishable characteristics for both seen and unseen classes. Firstly, the model is pretrained by a distance prediction loss to avoid overfitting. Then, the model only selects attributes of similar seen classes and makes sparse representations based on attributes for unseen classes, thereby overcoming negative transfer. After the model synthesizes pseudo-features for unseen classes, it disposes of the pseudo-feature outliers to improve the class discriminability. The pseudo-features are fed into a classifier of the model together with features of seen classes for GZSL classification. Experimental results on four benchmark datasets verify that the proposed DPFS has GZSL classification performance better than that in existing methods.

## 1. Introduction

Target classification and recognition have been dramatically improved with the development of deep learning technologies. Traditional deep learning methods rely heavily on large-scale labelled training datasets such as ImageNet [1]. However, some are infeasible in extreme cases without labelled samples of some classes [2]. To address it, zero-shot learning (ZSL), which imitates the process of human recognition, has been proposed to link seen classes (available in training datasets) and unseen ones (not available in training datasets) using auxiliary information (e.g., attributes [3] and word vectors [4]). Conventional ZSL methods only consider the recognition of unseen classes but neglect that of seen classes. It leads to the failure of simultaneous recognition of them [5]. Subsequently, generalized zero-shot learning (GZSL) [6] has been found to address it.

Most previous GZSL works are mainly divided into mapping-based approaches [7, 8] and hybrid approaches. The former learns a visual-semantic projection model trained with labelled samples. However, they are prone to overfitting due to limitation of labelled sample numbers and domain shift between disjointed seen classes and unseen classes [9], failing in unseen class classification. The latter, including generating-based approaches [10] and synthesis-based ones, has been proposed to alleviate overfitting. Generating-based approaches (e.g., generative adversarial networks (GANs) [11] and variational auto-encoders (VAEs) [12]) generate pseudo-features for unseen classes with prior semantic knowledge. However, they suffer from mode collapse [13] because it is challenging to train hybrid models. Unlike them, synthesis-based approaches [14–16] synthesize pseudo-features for unseen classes by using semantic information and seen class features. However, they suffer from negative transfer [17] and low-quality class discriminability [18].

In this paper, we propose a novel two-stage method of distinguishable pseudo-feature synthesis (DPFS) for GZSL tasks, as shown in Figure 1. Here, the embedding network and the preclassifier are jointly pretrained to extract distinguishable features for seen classes and simultaneously predict prototypes for unseen ones in stage 1. It ensures that the features of seen classes are well-kept and avoids overfitting effectively. Next, distinguishable pseudo-features of unseen classes are synthesized through the attribute projection module (APM) and the pseudo-feature synthesis module (PFSM) in stage 2. Here, for each unseen class, APM builds a sparse representation based on attributes to output a base vector. It only uses attributes of the base classes (i.e., the similar seen classes), thereby overcoming negative transfer. Furthermore, PFSM creates feature representations and synthesizes the pseudo-features by using the base class features, the base vectors and the unseen class attributes. The outliers of pseudo-features are disposed of to get distinguishable pseudo-features and improve the class discriminability. The distinguishable features are fed to the classifier to boost GZSL classification performance.

Our major contributions are summarized as follows:

1. We proposed a novel generalized zero-shot learning (GZSL) method of distinguishable pseudo-feature synthesis (DPFS). The proposed method can further improve GZSL classification performance compared with other state-of-the-art methods.
2. We pretrained our model by a well-designed distance prediction loss while predicting prototypes for unseen classes, thereby avoiding overfitting.
3. We only selected attributes of similar seen classes when making sparse representations based on attributes for unseen classes, thereby overcoming negative transfer effectively.
4. We screened the outliers of synthesized pseudo-features and disposed of them to further improve class discriminability.

## 2. Related Works

Mapping-based approaches can be traced back to early ZSL tasks [2–4, 9]. They learn a mapping function between visual features and semantic features by supervised learning. So, it is important to construct a feature-semantic loss function that can be used to train mapping model [19]. But early methods are prone to overfitting in GZSL tasks [7]. CPL [8] learned visual prototype representations for unseen classes to solve the problem. To obtain discriminative prototype, DVBE [20] used second-order graphical statistics, DCC [21] learned the relationship between embedded features and visual features, and HSVA [22] used hierarchical two-step adaptive alignment of visual and semantic feature manifolds. However, the prototype representation is constrained and does not correspond to actual features [10] due to domain shift. Different from these works, we propose a distance prediction loss, which constructs not only feature-attribute distance constraint of seen classes but also predicts unseen class prototypes under the guidance of a preclassifier. It keeps seen class features from disturbing the classification of unseen classes to avoid overfitting.

Generating-based approaches [23, 24], which utilize GANs and VAEs, have been widely applied to produce information about unseen classes and improve the prototype representation for GZSL tasks. They generate pseudo-features for unseen classes under the prior condition of semantic knowledge and random noise. LDMS [25], Inf-FG [26], and FREE [27] improved the generating strategy from aspects of discrimination loss, consistency descriptors, and feature refining. Besides, GCF [28] presented counterfactual-faithful generation to solve recognition rate imbalance between both seen classes and unseen ones. Although the strategies of generating-based methods are added to our proposed method, the use of simplex semantic information and the training difficulty [16] of GANs cause mode collapse.

Synthesis-based approaches [24, 29] integrate features and semantics of seen classes to enhance the feature diversity. SPF [15] designed a synthesis rule to guide feature embedding. TCN [14] exploited class similarities to build knowledge transfer from seen to unseen classes. To deal with the domain shift, LIUF [16] synthesized domain invariant features by minimizing the maximum mean discrepancy distance of seen class features. However, it would lead to negative transfer by mixing irrelevant class information. Different from the above mentioned, we only select the similar seen classes, instead of all seen classes, to finish knowledge transfer, thereby avoiding negative transfer caused by the mixing of irrelevant information. Then, we utilize distinguishable features extracted from the pretrained embedding network to apply to the pseudo-feature synthesis. Besides, we use a preclassifier to dispose of the outliers of synthesized components, thereby improving class discriminability. Unlike the method [24] of using synthesized elements from other domains, we only utilize the similar seen classes from this domain to overcome the unavailability of data from other domains.

## 3. Proposed Method

GZSL is more challenging than ZSL, which recognizes samples only from unseen classes, because GZSL needs to recognize samples from seen classes and unseen classes. Therefore, we propose the DPFS method to improve the theoretical basis of GZSL further and boost the classification performance. DPFS can synthesize distinguishable pseudo-features for unseen classes, and then use the pseudo-features to finish GZSL classification together with features of seen classes. In this chapter, we first define notations and definitions of GZSL, then outline the proposed method, including base class selection, distinguishable feature extraction, attribute projection, and distinguishable pseudo-feature synthesis. Finally, we provide the process of our training algorithm.

### 3.1. Mathematical Formulation

In GZSL tasks, suppose we have *S* seen classes *y*^*S*^ and *U* unseen classes *y*^*U*^, *y*^*S*^∩*y*^*U*^=∅. We give training dataset ∆^S^={*y*^*s*^(*x*_*i*_, *y*_*i*_) ∈ Ξ × y^S^}_*i*=1_^*n*_s_^ where *n*_s_ is the sample number, Ξ is visual space, *x*_*i*_ is a visual feature, and *y*_*i*_ is the class index of *x*_*i*_. The mapping function of the embedding network is denoted as *φ* : Ξ⟶*ς* where *ς* is latent space. The weight parameters of the embedding network, the preclassifier and the classifier are *θ*_en_, *θ*_pcls_, and *θ*_cls_, respectively. **A**^*S*^=[*a*_1_^*S*^,…, *a*_*S*_^*S*^] and **A**^*U*^=[*a*_1_^*U*^,…, *a*_*U*_^*U*^] are class-attribute matrices of seen classes and unseen classes, respectively. s and *u* are indexes of seen classes and unseen classes, *s* ∈ *y*^*S*^ and *u* ∈ *y*^*U*^, respectively.

GZSL methods learn a function *f*_GZSL_ : Ξ⟶*y*^*S*^ ∪ *y*^*U*^ with training dataset ∆^*S*^, and class-attribute matrices **A**^*S*^ and **A**^*U*^ to classify disjoint seen classes and unseen ones at the same time. After the training, both seen and unseen classes from testing datasets will be predicted by *f*_GZSL_.

### 3.2. Base Class Selection

For each unseen class, we only select the top *K* seen classes similar to the unseen classes to overcome negative transfer. Attributes of all base classes of unseen class *u* are with the closest distance to the attribute of the unseen class, which are as follows:

(1) $$\begin{array}{c} {Β}_{u}=\left\{1-\frac{a_{u}^{U}{∙a}_{s}^{S}}{\left\|a_{s}^{S}\right\|\left\|a_{u}^{U}\right\|}|s\in y^{S}\right\}\text{,} \end{array}$$

(2) $$\begin{array}{c} y_{u}^{B}=\left\{k|1-\frac{a_{u}^{U}∙a_{k}^{S}}{\left\|a_{u}^{U}\right\|\left\|a_{k}^{S}\right\|}\in topk\left(B_{u}\right)\right\}\text{,} \end{array}$$

where top*k*(∙) is an operator that sorts elements from small to large and selects indices of the top *K* elements. *y*_*u*_^*B*^ stones indices of the top *K* base classes, which are the first to the *K* th seen classes most similar to unseen class *u*.

### 3.3. Distinguishable Feature Extraction

In stage 1, we pretrain the embedding network and the preclassifier. It makes the embedding network extract distinguishable features for seen classes to build a relationship between classes and semantics, as shown in Figure 1. The attributes obtained by cognitive scientists [30] are the most commonly used semantic knowledge, and they are based on the high-level description of target objects specified by human beings [2]. We introduce the constraint of feature-attribute distance by imitating meta-learning [31], and build prototype representations, as shown in Figure 2. The customary way to construct the meta-learning task is called as *K*-way-*N*-shot [32], where *N* labelled samples in each of the *K* classes are provided in each iteration of the model training.

We randomly sample one unseen class and *K* seen classes per iteration. And, we set support set Σ={(*x*_*i*_, *y*_*i*_)*|y*_*i*_ ∈ Ψ^*S*^}_*i*=1_^*N*×*K*^ and query set Θ={(*x*_*i*_, *y*_*i*_)*|y*_*i*_ ∈ Ψ^*S*^}_*i*=*N*×*K*+1_^*N*×*K*+*Q*×*K*^. The visual features from Σ produce prototypes for seen classes through the embedding network are as follows:

(3) $$\begin{array}{c} c_{y_{i}}=\frac{\sum_{i=1}^{N}E_{\theta_{en}}\left(x_{i}\right)}{N}\text{,} \end{array}$$

where *x*_*i*_ is a visual feature from seen class *s* and *N* is the class number. Then, a feature-attribute distance (FAD) loss is constructed as follows:

(4) $$\begin{array}{c} \Lambda_{FAD}=\underset{\left(x_{i},y_{i}\right)\in \Theta }{\sum }\left({\left\|E_{\theta_{en}}\left(x_{i}\right)-c_{y_{i}}\right\|}_{2}^{2}+{\left\|c_{y_{i}}-a_{y_{i}}^{S}\right\|}_{2}^{2}\right)\text{.} \end{array}$$

Different from the meta-representation [33] restrained by the distance minimization of intraclass features, we act on the feature-attribute distance constraint to structure the meta-representation associating common characteristics between different attributes. After the constraint, features in latent space are pulled near their prototypes to ensure that the similar attracts and the dissimilarity repels each other. The prototype and the attribute from the same class are close to each other. Therefore, the features of seen classes in latent space can be regarded as the distinguishable features extracted from the embedding network.

To keep the embedding network from overfitting, the prototypes are predicted by features of their base classes. A component from the base class is denoted as follows:

(5) $$\begin{array}{c} v_{k}=E_{\theta_{en}}\left(choice\left(b_{k}\right)\right)\text{,} \end{array}$$

where choice(∙) is a choice operator, specifically choice(*b*_*k*_) means randomly choosing a visual feature of the *k* th similar base class from Ψ_*u*_^*B*^. A predicted prototype is denoted as follows:

(6) $$\begin{array}{c} {\tilde{c}}_{u}=\frac{\sum_{b_{k}\in \Psi_{u}^{B}}v_{k}+a_{u}^{U}}{K+1}\text{.} \end{array}$$

For each iteration, we build a prototype query set $\Theta^{U}={\left\{\left({\tilde{c}}_{u},u\right)|y_{i}\in \Psi^{U}\right\}}_{i=1}^{U}$. Then, a preclassification loss Λ_PC_ operating to pretrain the preclassifier is donated as follows:

(7) $$\begin{array}{c} \Lambda_{PC}=\underset{\left(x_{i},y_{i}\right)\in \Theta }{\sum }\log\;\left(P_{\theta_{pcls}}\left(y_{i}|E_{\theta_{en}}\left(x_{i}\right)\right)\right)-\underset{\left({\tilde{c}}_{u},u\right)\in \Theta^{U}}{\sum }\log\left(P_{\theta_{pcls}}\left(u|{\tilde{c}}_{u}\right)\right), \end{array}$$

where *p*(∙*|*∙) is a SoftMax function for the preclassification. Then, Λ_FAD_ and Λ_PC_ are summed to form distance prediction loss Λ_DP_ as follows:

(8) $$\begin{array}{c} \Lambda_{DP}=\Lambda_{FAD}+\Lambda_{PC}\text{.} \end{array}$$

We use the distance prediction loss to jointly pretrain the embedding network and the preclassifier. After that, seen classes will be classified, and unseen classes will be predicted preliminarily. It prevents trade-off failure between seen and unseen classes. Besides, features of seen classes will be extracted, and then used for unseen pseudo-feature synthesis.

### 3.4. Attribute Projection

Inspired by sparse coding, we make a sparse representation for each unseen class. We select attributes only from the base classes unlike the methods [14, 16] using all seen classes, to build attribute projections from seen to unseen classes. For unseen class *u*, the matrix of its attribute projection is denoted as follows:

(9) $$\begin{array}{c} M_{u}=\left[\begin{array}{ccc} a_{b_{1}}^{S} & \ldots & a_{b_{K}}^{S} \end{array}\right]\text{,} \end{array}$$

where *a*_*b*_1__^*S*^, *a*_*b*_*K*__^*S*^ ∈ Ψ_*u*_^*B*^. The attribute projection can represent the unseen class information by using sparse representation vector set {*m*_*u*_}_*u*=1_^*U*^. The objective function of the attribute projection is as follows:

(10) $$\begin{array}{c} m_{u}=\arg\underset{m_{u}}{\;\min}{\left\|a_{u}^{U}-M_{u}m_{u}\right\|}_{2}^{2}+\beta_{1}{\left\|m_{u}\right\|}_{1}+\beta_{2}{\left\|m_{u}\right\|}_{2}^{2}\text{,} \end{array}$$

where *β*_1_ and *β*_2_ are two regulation coefficients, *β*_1_, *β*_2_ > 0. The mixed regularizations of *L*1-norm and *L*2-norm have the advantages of sparsity and trade-off between deviation and variance [34]. Both *β*_1_ and *β*_2_ are set as 0.4 with appropriate generality. The objective function is optimized by the optimal local condition of Karush-Kuhn-Tucker [35] where *m*_*u*_ are non-negative. We normalize *m*_*u*_ by using the following equation:

(11) $$\begin{array}{c} m_{u}=\frac{m_{u}}{\left\|m_{u}\right\|}\text{.} \end{array}$$

Then, we treat *m*_*u*_ as the base vector. The attribute projection provides a vital item for the pseudo-feature synthesis, as shown in Figure 3.

### 3.5. Distinguishable Pseudo-Feature Synthesis

For unseen class *u*, we randomly choose a feature from each of its base classes to construct an embedding matrix $\left[\begin{array}{ccc} v_{1} & \cdots & v_{K} \end{array}\right]$. The base vectors are utilized for weighting the chosen features that are embedded into the attribute projection, as shown in Figure 3(a). Then, a feature representation is formulated as follows:

(12) $$\begin{array}{c} \tilde{v}=\left(1-\gamma \right)\left[\begin{array}{ccc} v_{1} & \cdots & v_{K} \end{array}\right]m_{u}+\gamma a_{u}^{U}\text{,} \end{array}$$

where *γ* is a weighting coefficient (*γ* ∈ [0,1]). However, the feature representation only integrated with features of the base classes may be scattered and produce outliers of candidate pseudo-features, as shown in Figure 3(b). Therefore, attribute information is integrated into the feature representation to synthesize candidate pseudo-features, as shown in Figure 3(c).

To dispose of the outliers, we screen them by the following equation:

(13) $$\begin{array}{c} f\left(\tilde{v}\right)=\left\{\begin{array}{c} 0,\max_{s\in \Psi^{S}}P_{\theta_{pcls}}\left(s|\tilde{v}\right)\geq \tau \text{,}\\ 1,otherwise\text{,} \end{array}\right. \end{array}$$

where *τ* is creditability threshold (*τ* ∈ [0,1]). The preclassifier acts as an operator of the outlier disposing. It screens and reserves the credible pseudo-features satisfying $f\left(\tilde{v}\right)=1$ to get distinguishable pseudo-features of unseen classes, as shown in Figure 3(d). After the operations of the attribute projection and the pseudo-feature synthesis, the synthesized features integrated with the information of the similar base classes and unseen classes have separability characteristics.

### 3.6. Train and Inference

We conduct the DPFS model training. Algorithm 1 shows the pseudo-code of the DPFS training algorithm. The algorithm mainly includes two-cycle structures because DPFS is a two-stage method. Firstly, the sequence structure from lines 1 to 2 performs the attribute projection to get the base vector for each unseen class. Next, the first cycle from lines 3 to 9 performs the embedding module pretraining to extract distinguishable features of seen classes. Then, the second cycle from lines 10 to 15 performs the classifier training for GZSL tasks. In each iteration of the classifier training, we randomly select a certain number of the whole samples from training samples and synthesized pseudo-feature samples, where the number of the selected whole samples is *N*_*w*_. Here, the proportion of the pseudo-feature samples in the whole samples is set as *η*. After each iteration, the classifier is adopted for evaluation.

## 4. Experimental Results

### 4.1. Datasets

The DPFS model is evaluated on four widely datasets as evaluating benchmarks, i.e., Animals with Attributes 2 (AWA2 [6]), aPascal & Yahoo (aPY [36]), Caltech UCSD Birds 200 (CUB [37]), and SUN Attribute (SUN [38]). AWA2 and aPY are coarse-grained datasets and aPY includes a higher proportion of unseen classes than AWA2. CUB and SUN are fine-grained datasets, especially SUN, with more whole classes and fewer training samples per class than CUB.  Table 1 summarizes the statistics of the four evaluating benchmarks.

### 4.2. Implementation Details

We conduct ResNet-101 [39] as a backbone based on a convolutional neural network. Visual features are extracted from the output of the final avg-pooling layer after the backbone is pretrained on ImageNet [1].  Figure 4 shows the network structures of the DPFS model including the embedding network, the preclassifier and the classifier. The embedding network is composed of three fully connected (FC) layers, and the back of each layer is connected to a ReLU activation function for nonlinear activation. Both the preclassifier and the classifier have the same modules. Their modules are composed of two FC layers and the output dimensions equal the total number of all classes. For the four benchmarks, the middle layer dimension of the classifier is 512 for AWA2 and aPY, and 1024 for CUB and SUN, respectively.

Our model is coded in PyTorch and runs on GeForce RTX 2080 Ti. It is trained by an adaptive moment estimation (Adam) [40] optimizer. During the embedding module pretraining, sample numbers of each class in both the support set and the query set, *N* and *Q*, are set as 4 for AWA2, aPY, and CUB, and 2 for SUN, respectively. The learning rate of our model is 10^−4^. During the classifier training, the number of the whole selected samples, *N*_*w*_ is set as 1000. The classifier is trained with a learning rate of 10^−4^ and the embedding module is fine-tuned with a learning rate of 10^−6^. Besides, four additional hyper-parameters, the proportion of pseudo-feature samples *η*, creditability threshold *τ*, number of base classes *K*, and weighting coefficient *γ* will be discussed later in the hyper-parameter sensitivity chapter. Samples from training datasets are used to train our model by supervised learning. And samples from the testing datasets are used to evaluate GZSL classification performance of our model.

The accuracies of average seen classes (*As*) and average unseen classes (*Au*) are computed based on the universal evaluation protocols [6].

(14) $$\begin{array}{c} As=\frac{1}{\left|\Psi^{S}\right|}\underset{y\in \Psi^{S}}{\sum }\frac{\#\;correct\;pre\;di\;ctions\;in\;y}{\#\;samples\;in\;y}\text{,} \end{array}$$

(15) $$\begin{array}{c} Au=\frac{1}{\left|\Psi^{U}\right|}\underset{y\in \Psi^{U}}{\sum }\frac{\#\;correct\;pre\;di\;ctions\;in\;y}{\#\;samples\;in\;y}\text{.} \end{array}$$

We evaluate the simultaneous classification accuracy of both seen and unseen classes by computing harmonic mean *H* as follows:

(16) $$\begin{array}{c} H=\frac{2\times As\times Au}{As+Au}\text{,} \end{array}$$

*H* is regarded as the most crucial criterion to measure the GZSL classification performance.

### 4.3. Hyper-Parameter Sensitivity

There are four hyper-parameters including the proportion of pseudo-feature samples *η*, creditability threshold *τ*, number of base classes *K*, and weighting coefficient *γ*. We discuss the sensitivity of the hyper-parameters because proper hyper-parameters give our model extra reliability and robustness.

Proportion *η* controls the frequencies of obtaining information from seen classes and unseen ones. Higher *η* provides the classifier with more opportunities to learn the characteristics of unseen classes.  Figure 5 shows GZSL classification performance under different *η* on the four benchmarks. We set *η* within the range from 0.7 to 0.97 and select the proper *η* value according to the optimal GZSL performance.

*As* will decrease slowly while *Au* and *H* will increase until reaching a peak along with the increase of *η* in most cases. This result reveals that DPFS can provide more balanced GZSL performance by adjusting *η*. The decreasing ratio of *As* will increase after *Au* and *H* reach the peak. It indicates a proper selection of *η* is necessary to solidify seen class classification. When *H* reaches the peak, *η* is different on the four benchmarks. The value depends on the granularity of training samples. In general, the value on the benchmarks with a few training samples (such as SUN) should be lower than that on the benchmarks with multitraining samples (such as AWA2), and the value on the benchmarks with a higher proportion of unseen classes (such as aPY and CUB) should be higher. Therefore, we set *η* = 0.85 for AWA2, *η* = 0.94 for aPY, *η* = 0.91 for CUB, and *η* = 0.76 for SUN.

Creditability threshold *τ* controls the effect of the outlier disposing.  Figure 6 shows the performance under different *τ* on the four benchmarks. We set *τ* within the range of 0.7 to 0.95. This result reveals that *As* will decrease and *Au* will increase along with the increase of *τ* in most cases. Meanwhile, *H* will increase until reaching a peak. When the range of *τ* is 0.8 to 0.9, *H* will reach the peak, and the classification accuracy will be the best. It indicates proper *τ* can prevent the outliers from interfering with seen class classification while maintaining unseen class classification. Therefore, we set *τ* = 0.85 on all the four benchmarks.

Numbers of base classes and weighting coefficient, *K* and *γ*, concurrently control the pseudo-feature synthesis simultaneously.  Figure 7 shows the *H* heatmap results of the performance under different *K* and *γ* values on the four benchmarks. The range of *K* is set from 3 to 9 for AWA2 and CUB, from 6 to 12 for aPY, and from 2 to 8 for SUN, respectively. The range of *γ* is set from 0 to 0.4.

The result reveals that *N* has a more significant impact than *γ* on *H*. *H* will increase first and then reduce along with the increase of *N*. It indicates that an appropriate integration with the similar seen classes will achieve outstanding classification accuracy, but an over-integration will degrade the classification accuracy because it mixes information of irrelevant classes. According to the performance on the four benchmarks, *N* making *H* reach peak depends on the granularity of training samples. In general, *N* on the benchmarks with a few training samples (such as CUB and SUN) should be lower than that on the benchmarks with multitraining samples (such as AWA2), and *N* on the benchmarks with the higher proportion of unseen classes (such as aPY) should be higher. So, we set *N* = 5 for AWA2, *N* = 9 for aPY, *N* = 6 for CUB, and *N* = 3 for SUN.

The result also reveals that when *N* is fixed, *H* will also increase first and then reduce along with the increase of *γ* in most cases. It indicates that weighting a certain proportion of attributes will improve the classification accuracy and the proper introduction of attribute information can raise the performance of our model. Therefore, we set *γ* = 0.2 for AWA2, *γ* = 0.3 for aPY, *γ* = 0.1 for CUB, and *γ* = 0.35 for SUN.

### 4.4. Performance Results

Table 2 shows GZSL classification performance results compared with existing state-of-the-art approaches and the proposed DPFS. The existing approaches contain the mapping-based, the generating-based, and the synthesis-based approaches, which are marked with †, ⸶, and ⸷, respectively. Among these, the results show that DPFS gains the best performance on AWA2, CUB, and SUN, and achieves the second performance on CUB. Compared with the mapping-based approaches, DPFS is superior to DCC by 5.5% on aPY, and DVBE by 4.8%, 2%, and 5.4% on AWA2, CUB, and SUN, respectively. Compared with the generating-based approaches, DPFS is superior to FREE by 4.7% on AWA2, LDMS by 4.9% on aPY, and GCF by 3.9% on SUN, respectively. And compared with the synthesis-based approaches, DPFS is superior to LIUF by 1.6%, 1.1%, 6%, and 3.2% on AWA2, aPY, CUB, and SUN, respectively. DPFS significantly improves *Au* and avoids overfitting.

DPFS is superior to most mapping-based approaches in the aspects of *Au* and *H*, especially on SUN. It indicates that DPFS has a more vital learning ability on the benchmarks with a few training samples. And DPFS shows significant improvement of *As*, *Au*, and *H*, especially compared to generating-based approaches on aPY. It explains that DPFS makes full use of the feature information of seen classes and the attribute information, thereby solving the difficulty of classifying the higher proportion of unseen classes and avoiding mode collapse.

DPFS also experiments on the four benchmarks for conventional ZSL tasks, where only the synthesized pseudo-feature samples are fed into the classifier.  Table 3 shows ZSL classification performance results. We observe that DPFS overperforms existing methods on AWA2, aPY, and SUN, which can also verify that the synthesized pseudo-features have distinguishable characteristics.

We further demonstrate the advantage of DPFS over SPF and LIUF. We imitate SPF and LIUF, replacing the strategy of our pseudo-feature synthesis with the synthesis strategies of SPF and LIUF to form the reference methods, D-SPF and D-LIUF, respectively. Meanwhile, the stages of the embedding module pretraining and classifier training of D-SPF and D-LIUF are the same as those of DPFS.  Table 4 shows the comparison results among D-SPF, D-LIUF, and DPFS. DPFS gains prominent advantages over D-SPF because the optimized attribute projection can embed and project features of seen class into features of unseen class more accurately, to improve class discriminability. DPFS also has apparent advantages over D-LIUF especially on CUB and SUN. DPFS eliminates the irrelevant classes, so it suppresses negative transfer. In addition, DPFS introduces the attribute weighting in equation (12) and the outlier disposing in equation (13), to decrease the confusion between classes. So, DPFS is superior to D-SPF and D-LIUF in classification.

### 4.5. Ablation Results

We conducted ablative experiments to illustrate the influence of different tactics in DPFS. The tactics contain the embedding module pretraining (mpt), the outlier disposing (odi) in equation (13), and the preclassification loss (pc) in equation (7).  Table 5 shows the results of ablation experiments. Four ablated methods, PFS, DPFS-1, DPFS-2, and DPFS-3 are all validated. PFS is to remove all the tactics. DPFS-1, which pretrains the model only by the feature-attribute distance loss in equation (4), is to add the mpt tactic. DPFS-2 is to add both the mpt and odi tactics. And DPFS-3, which pretrains the model by the distance prediction loss in equation (8), is to add both the tactics of mpt and pc.

It is important to add the mpt tactic for extracting some common characteristics between seen classes and unseen ones because it improves prototype representations and eliminates the domain shift. Therefore, DPFS-1 performs obvious progress compared with PFS. PFS-1 is superior to PFS by 8.6% on AWA2, 8.3% on aPY, 9.3% on CUB, and 9.3% on SUN. On this foundation, DPFS-2 adopts the odi tactic to eliminate the outliers of candidate pseudo-features. It boosts the performance on parts of benchmarks. PFS-2 is superior to PFS-1 by 0.9% on AWA2, and 0.4% on aPY, respectively. DPFS-3 adopts the pc tactic to predict prototypes for unseen classes before the classifier training, thus improving the classification performance. PFS-3 is superior to PFS-1 by 2.9% on AWA2, 6.6% on aPY, 1.5% on CUB, and 2.4% on SUN, respectively. DPFS can cohere all the features in the same class and therefore avoid outlier interference. Thus, DPFS adopting the three auxiliary tactics at the same time makes the best progress in *H* on the four benchmarks. And, DPFS is superior to PFS-3 by 1.7% on AWA2, 2% on aPY, 1.7% on CUB, and 2.6% on SUN.

We visualize features from the embedding module by t-SNE [41] to further show the tactic effect on the AWA2 benchmark for GZSL tasks.  Figure 8 shows the visualization results. We find that DPFS can improve the distinguishability of unseen classes. Meanwhile, it can also maintain the distinguishability of seen classes according to the comparison results between Figures 8(a), 8(c) and 8(b), and 8(d). Considering that existing methods [18, 26] do not visualize all features of both seen and unseen classes, we visualize all the output features of testing samples from PFS and DPFS in Figures 8(e) and 8(f), respectively. It is obvious that the classes characterized by the output features from DPFS is more separable than those characterized by the output features from the PFS. DPFS eliminates the confusion between classes and improves feature distinguishability, thus achieving a better multiclass classification accuracy. Both seen and unseen classes satisfy the characteristics of intraclass gather and interclass separability. Therefore, DPFS can effectively eliminate the domain shift.

## 5. Discussion

Based on the results above, our model was trained and evaluated on four benchmark datasets. Our method selected the optimal hyper-parameters for different benchmarks to achieve the best GZSL classification performance compared with most existing methods. Especially on the benchmarks with a few training samples or with a higher proportion of unseen classes, DPFS gained the superior performance because it can use the information of features and attributes appropriately and avoid mode collapse. Compared with existing synthesis-based models similar to DPFS, DPFS can eliminate the introduction of irrelevant classes and suppress negative transfer. It can also synthesize candidate pseudo-features and dispose of the outliers to improve class discriminability.

Furthermore, our model was also trained and evaluated for ZSL tasks and outperformed competing ZSL methods on most benchmarks. Besides, we conducted the ablation experiments of DPFS and further explained the performance gain of each tactic. Distinguishable features can be extracted and the GZSL performance can be improved with the embedding module pretraining tactic. On this basis, adding the preclassification tactic can predict prototypes for unseen classes before the classifier training, thereby improving the performance and avoiding overfitting. The tactic of the outlier disposing can further enhance the performance. These are the foundation that outperforms the competing GZSL methods. The visualization results have demonstrated that DPFS has the distinguishability characteristics of both seen and unseen classes.

## 6. Conclusion

This paper proposed a novel distinguishable pseudo-feature synthesis (DPFS) method for GZSL tasks. It included the procedures of base class selection, distinguishable feature extraction, attribute projection, feature representations, and outlier disposing. These procedures can realize the initialization, the connection, and the weight updating of the DPFS model. Therefore, the model can synthesize distinguishable pseudo-features with attributes of unseen classes and features of similar seen classes. Experimental results showed that DPFS achieved the GZSL classification performance better than existing methods. It indicated DPFS significantly improved class discriminability and restrained negative transfer, and DPFS also effectively eliminated the domain shift and the confusion between classes. In the future, we will synthesize more distinguishable features of unseen classes by integrating more auxiliary information, such as statistical features and knowledge graphs, to extend our method into other applications.

## Figures and Tables

**Figure 1:** Illustration of DPFS. (a) DPFS consists of an embedding network, an attribute projection module (APM), a pseudo-feature synthesis module (PFSM), a preclassifier and a classifier. In stage 1, the embedding network and the preclassifier are jointly pretrained to extract distinguishable features for seen classes. In stage 2, the network synthesizes distinguishable pseudo-features for unseen classes through APM and PFSM. Then, the features and the pseudo-features are fed into the classifier for GZSL tasks. (b) APM Details. APM builds sparse representations based on attributes. (c) PFSM Details. PFSM creates feature representations and synthesizes distinguishable pseudo-features with the selected features, the base vectors, and the unseen class attributes. The outliers of candidate pseudo-features are disposed of to get distinguishable pseudo-features.

**Figure 2:** Illustration of feature-attribute distance constraint. For example, the unseen class is a bobcat and its base classes are leopard, fox and wolf.

**Figure 3:** Illustration of pseudo-feature synthesis. (a) Attribute projection. (b) Results after the attribute projection. (c) Results after the attribute weighting. (d) Results after the outlier disposing.

**Figure 4:** Illustration of network structures of the embedding network, the preclassifier and the classifier. In the embedding network, the dimensions of the input and the output features are marked on the left side and the right side of the FC layers, respectively. “V-D”, “S-D”, “C-D”, and “Dim” are the dimensions of visual features, the output features of the embedding network, the class number, and the middle layer dimension of the preclassifier/classifier, respectively.

**Figure 5:** Results of classification under different *η* on (a) AWA2, (b) aPY, (c) CUB, and (d) SUN.

**Figure 6:** Accuracy of classification under different *τ* on (a) AWA2, (b) aPY, (c) CUB, and (d) SUN.

**Figure 7:** Four *H* heatmaps under different *N* and *γ* on (a) AWA2, (b) aPY, (c) CUB, and (d) SUN. Each row and each column denote the results of different *N* and *γ*, respectively. In each heatmap, brighter colour represents greater *H*.

**Figure 8:** T-SNE visualization of features in 40 seen classes (a, b), 10 unseen classes (c, d) and all 50 classes (e, f) on AWA2 by PFS (a, c, e) and DPFS (b, d, f) in GZSL tasks. Different colours denote different classes. It is obvious that DPFS can provide more separable classes.

**Algorithm 1:** DPFS training algorithm

**Table 1:** Statistics of the four benchmark datasets.

Dataset	Number of classes			Attribute	Number of samples			
	Seen	Unseen	Total		Training	Seen testing	Unseen testing	Total
AWA2	40	10	50	85	23527	5882	7913	37322
APY	20	12	32	64	5932	1483	7924	15339
CUB	150	50	200	312	7057	1764	2967	11788
SUN	645	72	717	102	10320	2580	1440	14340

**Table 2:** Quantitative comparisons of average per-class GZSL classification accuracy (%).

Method		AWA2			aPY			CUB			SUN		
		*As*	*Au*	*H*	*As*	*Au*	*H*	*As*	*Au*	*H*	*As*	*Au*	*H*
†	LATEM [9]	77.3	11.5	20.0	73.0	0.1	0.2	57.3	15.2	24.0	28.8	14.7	19.5
	DEM [19]	86.4	30.5	45.1	75.1	11.1	19.4	54.0	19.6	13.6	34.3	20.5	25.6
	CPL [8]	83.1	51.0	63.2	73.2	19.6	30.9	58.6	28.0	37.9	32.4	21.9	26.1
	DVBE [20]	70.8	**63.6**	67.0	58.3	32.6	41.8	60.2	53.2	56.5	37.2	45.0	40.7
	DCC [21]	82.9	55.1	66.2	74.8	34.4	47.2	57.7	46.5	51.5	41.0	33.1	36.6
	HSVA [22]	79.3	57.8	66.9	—	—	—	59.5	51.9	55.5	39.0	48.6	43.3

†	SEZEL [23]	68.1	58.3	62.8	—	—	—	53.3	41.5	46.7	30.5	40.9	34.9
	DUET [10]	**90.2**	48.2	63.4	55.6	21.8	31.3	**80.1**	39.7	53.1	—	—	—
	Inf-FG [26]	63.4	58.3	60.7	—	—	—	57.0	45.8	50.8	37.1	44.7	40.5
	LDMS [25]	71.8	60.9	65.9	66.3	37.4	47.8	61.6	48.0	53.9	36.2	45.6	40.3
	FREE [27]	75.4	60.4	67.1				59.9	55.7	57.7	37.7	44.8	40.9
	GCF [28]	75.1	60.4	67.0	56.8	37.1	44.9	59.7	**61.0**	**60.3**	37.8	47.9	42.2

†	SPF [15]	60.9	52.4	56.3	—	—	—	63.4	30.2	40.9	**59.0**	32.2	41.6
	TCN [14]	65.8	61.2	63.4	64.0	24.1	35.1	52.0	52.6	52.3	37.3	31.2	34.0
	LIUF [16]	83.5	60.6	70.2	79.1	38.2	51.6	54.0	51.2	52.5	40.4	45.7	42.9
	**DPFS**	87.3	61	**71.8**	**83.0**	**38.6**	**52.7**	63.8	54.0	58.5	43.0	**49.6**	**46.1**

**Table 3:** Quantitative comparisons for the ZSL tasks.

Method	AWA2	aPY	CUB	SUN
LATEM [9]	55.8	35.2	49.3	55.3
SJE [4]	61.9	32.9	53.9	53.7
TVN [5]	68.8	41.3	58.1	60.7
CPL [8]	72.7	45.3	56.4	62.2
SEZSL [23]	69.2	—	59.6	63.4
ZVG [12]	69.3	37.4	54.8	59.4
HSVA [22]	—	—	62.8	63.8
DUET [10]	72.6	41.9	**72.4**	—
Inf-FG [26]	68.3	—	58.0	61.1
LDMS [25]	72.9	43.7	58.4	59.4
TCN [14]	71.2	38.9	59.5	61.8
LIUF [16]	72.4	59.3	43.7	63.3
DPFS	**73.9**	**61.4**	68.0	**66.8**

**Table 4:** Quantitative comparisons among D-SPF, D-LIUF, and DPFS.

Method	AWA2			aPY			CUB			SUN		
	*As*	*Au*	*H*	*As*	*Au*	*H*	*As*	*Au*	*H*	*As*	*Au*	*H*
D-SPF	81.3	55.4	65.9	64.5	32.9	43.5	**70.8**	44.0	54.3	**45.3**	42.4	43.8
D-LIUF	86.1	60.4	71.0	82.5	36.2	50.3	58.7	51.8	55.0	42.4	46.4	44.3
DPFS	87.3	61.0	71.8	83.0	38.6	52.7	63.8	54.0	58.5	43.0	49.6	46.1

**Table 5:** Ablation results on DPFS.

Method	Mpt	Odi	Pc	AWA2	aPY	CUB	SUN
				*H*	*H*	*H*	*H*
PFS				58.6	35.8	46.0	31.8
DPFS-1	√			67.2(+8.6)	44.1(+8.3)	55.3(+9.3)	41.1(+9.3)
DPFS-2	√	√		68.1(+9.5)	44.5(+8.7)	55.2(+9.2)	40.8(+9.0)
DPFS-3	√		√	70.1(+11.5)	50.7(+14.9)	56.8(+10.8)	43.5(+11.7)
DPFS	√	√	√	71.8(+13.2)	52.7(+16.9)	58.5(+12.5)	46.1(+14.3)

## Data Availability

The dataset AWA2 can be downloaded from https://cvml.ist.ac.at/AwA2/ or https://academictorrents.com/details/1490aec815141cdb50a32b81ef78b1eaf6b38b03. The other three datasets, aPY, CUB, and SUN can also be downloaded from https://vision.cs.uiuc.edu/attributes/, http://www.vision.caltech.edu/datasets/cub_200_2011/, and https://www.cnblogs.com/GarfieldEr007/p/5438417.html, respectively.
